# HMGCS2 silencing attenuates high glucose-induced in vitro diabetic cardiomyopathy by increasing cell viability, and inhibiting apoptosis, inflammation, and oxidative stress

This article has been retracted.

**DOI:** 10.1080/21655979.2022.2063222

**Published:** 2022-05-04

**Authors:** Donglin Chen, Xiang Ruan, Yu Liu, Yan He

**Affiliations:** a Department of General Geriatrics Division, The First Affiliated Hospital of Guangxi Medical University, Nanning, Guangxi, China; b Department of Cardiology, The People’s Hospital of Guangxi Zhuang Autonomous Region, Guangxi Academy of Medical Sciences, Nanning, Guangxi, China

**Keywords:** Diabetic cardiomyopathy, bioinformatics, HMGCS2, apoptosis, inflammation, oxidative stress

## Abstract

Diabetic cardiomyopathy (DCM) is a diabetic mellitus-related complications and progression of DCM may eventually lead to heart failure, while mechanisms related to DCM pathophysiology remain unclear. The study was undertaken to identify possible hub genes associated with DCM progression through bioinformatics analysis and to validate the role of 3-hydroxy-3-methylglutaryl-CoA synthase 2 (HMGCS2) in DCM progression using a cellular model of high glucose (HG)-induced DCM. The common differentially expressed genes (DEGs) between GSE173884 and GSE161827 were used for PPI network analysis. Our results identified 17 common DEGs between GSE173384 and GSE161827. Further analysis of the protein–protein interaction network identified nine hub genes and HMGCS2. The in vitro functional assays showed that HG induced up-regulation of HMGCS2, suppressed cardiomyocyte viability, enhanced apoptosis, inflammation, and oxidative stress of cardiomyocytes. Gain-of-function assays showed that HMGCS2 overexpression reduced cell viability, increased apoptosis, caspase-3/-9 activity, up-regulated interleukin (IL)-1β, IL-6 and tumor necrosis factor-α (TNF-α) expression, decreased superoxide dismutase (SOD), catalase (CAT) and glutathione peroxidase expression, increased malondialdehyde (MDA) content, and reactive oxygen species (ROS) level but inhibited total antioxidant activity, SOD activity, CAT activity, and glutathione content in cardiomyocytes. Rescue experiments demonstrated HMGCS2 silence attenuated HG-induced decrease in cardiomyocyte viability and increase in cardiomyocyte apoptosis, inflammation, and oxidative stress. All in all, our study identified HMGCS2 as a hub gene in DCM pathophysiology and further functional studies indicated that HMGCS2 may aggravate DCM progression by reducing cardiomyocyte viability, increasing cardiomyocyte apoptosis, and promoting inflammation and oxidative stress in cardiomyocytes.

## Highlights

- HMGCS2 was up-regulated in the heart tissues from the diabetic mice.
- High glucose induced up-regulation of HMGCS2, suppressed cardiomyocyte viability, enhanced apoptosis, inflammation and oxidative stress of cardiomyocytes.
- HMGCS2 overexpression promoted cardiomyocyte apoptosis, inflammatory response and oxidative stress.
- HMGCS2 silence attenuated HG-induced decrease in cardiomyocyte viability and increase in cardiomyocyte apoptosis, inflammation and oxidative stress.

## Introduction

Diabetic cardiomyopathy (DCM) is a frequently occurring complication in diabetic mellitus (DM) and is featured by ventricular mass elevation and persistent diastolic disturbance [1–6]. The progression of DCM can be caused by complicated factors such as mitochondria dysfunction, increased inflammation, hyperglycemia, and insulin resistance, which may impair heart function and eventually lead to heart failure [7–9]. Though great improvements have been made in the treatment of DCM, the underlying molecular mechanism involved in DCM development remains unclear. There is growing evidence suggesting that chronic hyperglycemia and lipid disorders can induce excessive production of reactive oxygen species (ROS) in diabetic hearts. Increased ROS could induce oxidative damage on the heart tissues [10,11]. Thus, how to counteract the excessive production of ROS may be a good strategy for the management of DCM.

Recent advances into high throughput profiles of genomes have provided researchers with effective tools to decipher the complex signaling pathways in various pathogenic conditions, including diabetic cardiomyopathy. Using the RNA-sequencing technology, researchers identified a novel long non-coding RNA (lncRNA) NONRATT007560.2 that can regulate high glucose-induced apoptosis and oxidative stress [12]. Microarray profiling studies also decipher the actions of miR-200b-3p/mRNA-CD36 modulates in DCM [13]. Studies also performed circular RNA profiling of the heart tissues from the diabetic mice and identified 58 differentially expressed circular RNAs that may be associated with the early-stage DCM [14]. Ju et al. showed that changes in N6-methyladenosine modification modulate DCM by reducing myocyte hypertrophy and myocardial fibrosis [15]. Recent study revealed Daw1, AK089884, G730013B05Rik, BC038927, 2700054A10Rik as key lncRNAs in DCM [16]. Studies also performed analysis using dataset GSE62203 and identified five potential biomarkers for DCM prognosis [17]. In this regard, using high throughput profiling methods to explore molecular mechanisms involved in DCM is an effective way to identify novel biomarkers associated with DCM.

In this study, we performed analysis using microarray datasets (GSE173884 and GSE161827) and extracted the differentially expressed genes (DEGs) in heart tissues with and without DCM. Based on DEGs, we constructed a protein–protein interaction (PPI) network and aimed to screen key genes. Furthermore, one of the hub genes was verified for its role in DCM by using the in vitro cellular functional assays. The present study may reveal some novel aspects of the DEGs in regulating DCM. The study workflow was demonstrated in Figure 1.

**Figure 1.** Diagram of the workflow in this study.

## Materials and methods

### Identification of common DEGs between collected datasets

Microarray datasets for GSE173884 and GSE161827 were extracted from the GEO website. For GSE173884 analysis, gene expression profiles from DCM heart of db/db mice and normal hearts of wild-type mice were performed using GPL24247 Illumina NovaSeq 6000, and DEGs in the DCM hearts compared to normal hearts were extracted using GREIN-iLINCS [18] with |log fold change (FC)| >1.5 and P <0.05. For GSE161827 analysis, gene expression files from DCM heart of four mice fed a high-fat, high-sucrose diet and normal hearts of four mice fed with a control diet were performed using GPL19057 Illumina NextSeq 500, and DEGs in the DCM hearts compared to normal hearts were extracted using GREIN-iLINCS [18] with |log FC| >1.5 and P <0.05. DEGs in GSE173884 and GSE161827 were visualized using volcano plots; the common DEGs between GSE173884 and GSE161827 were visualized using Venn diagram.

### PPI network construction and submodule extraction

Common DEGs extracted from GSE173884 and GSE161827 were used to generate a PPI network based on the STRING tool [19]. The generated PPI network detailed with gene interactions was imported into Cytoscape software, and the network was visualized by this software. Furthermore, hub genes were determined from the PPI network by using the Cytohubba tool to generate the key submodule.

### Cell culture, high glucose treatment, plasmid, and siRNA transfection

Rat cardiomyocytes (H9C2 cell line) were from ATCC company (Manassas). H9C2 cells were grown in DMEM (Sigma) supplemented with 10% fetal bovine serum (Sigma) with 5% CO_2_-air 37°C. For the high glucose (HG) treatment, H9C2 cardiomyocytes were incubated with 30 mM glucose (duration = 48 h). In terms of osmotic control, H9C2 cardiomyocytes were incubated with 30 mM mannitol (duration = 48 h). For the blank group, cells were treated with culture medium. Then, H9C2 cells were harvested and processed for downstream assays.

The 3-hydroxy-3-methylglutaryl-CoA synthase 2 (HMGCS2)-overexpressing vector was generated from inserting HMGCS2 into pcDNA3.1 plasmid (RiboBio), and blank pcDNA3.1 was used as negative control. HMGCS2 siRNA was synthesized by RiboBio and scrambled siRNA for HMGCS2 was used as negative control (si-NC). Cardiomyocytes transfection with plasmids or siRNAs was carried out by using Lipofectamine 2000 reagent (Invitrogen). Then, H9C2 cells were harvested and processed for downstream assays.

### Quantitative real-time PCR (qRT-PCR)

RNA from cardiomyocytes were harvested using TRIzol LS reagent (Invitrogen). Traces of genomic DNA contamination were cleared by RNase-free DNase (Ambion). Total RNA was reverse-transcribed to cDNA using Super-Script II (Invitrogen), and target genes were amplified using the standard RT PCR kit (Applied Biosystems). The amplification was performed in real-time PCR systems (Applied Biosystems). Gene expression by qRT-PCR was calculated after normalizing by GAPDH using the comparative Ct method. The primers were shown Supplemental Table S1.

### Cell Counting Kit-8 (CCK-8) assay

Cardiomyocyte viability was assessed by the CCK-8 assay kit (Beyotime). Briefly, cardiomyocytes received different interventions were plated into 96-well plates and were subjected to CCK-8 solution incubation for 2.5 h at 37°C. The absorbance at 450 nm wavelength was used as the index for cardiomyocyte activity.

### Terminal deoxynucleotidyl transferase dUTP nick end labeling (TUNEL) assay

Cardiomyocytes with different treatments were fixed with 4% paraformaldehyde and permeabilized with 0.1% Triton X-100. Cardiomyocyte apoptosis was detected by the In Situ Cell Death Detection Kit (Roche, Mannheim, Germany) according to the manufacturer’s protocol [20].

### Caspase-3 and caspase-9 activity assay

H9C2 cells with different interventions were lysed, and lysates were collected according to manufacturer’s protocol [21]. The caspase-3 and caspase-9 activity of H9C2 cell lysates were assessed by Caspase 3 Fluorimetric Assay Kit and Caspase 9 Fluorimetric Assay Kit, respectively (Beyotime), with a FLUOstar Optima plate reader.

### Total antioxidant

Cardiomyocyte antioxidant activity was determined by the Total Antioxidant Capacity Assay Kit (Beyotime) [22]. Briefly, cardiomyocytes with different interventions were lysed, and lysates were indicated with 2,2ʹ-azino-bis- (3-ethylbenzthiazolin-6-ammonium sulfonate followed by measuring antioxidant activity with determining absorbance at 374 nm.

### Superoxide dismutase (SOD) activity

Cardiomyocyte SOD activity was determined by the SOD activity kit (Beyotime) [23]. Briefly, cardiomyocytes that received different interventions were lysed, and the lysates were 2-(4-iodophenyl)-3-(4-nitrophenol)-5- phenyltetrazolium chloride followed by measuring the SOD activity with determining absorbance at 505 nm.

### Catalase (CAT) activity and glutathione (GSH) content

Cardiomyocyte CAT activity and GSH content were determined by the corresponding CAT activity kit (Thermo Fisher Scientific) and GSH assay kit (Thermo Fisher Scientific) according to the manufacturer’s protocol [24,25].

### Malondialdehyde (MDA) content

Cardiomyocyte MDA content was assessed by an MDA assay kit (Sigma) [26]. Briefly, cardiomyocytes that received different interventions were homogenized followed by mixing with thiobarbituric acid reagent. The mixed solution was boiled for 15 min followed by centrifugation at 4000 rpm for 8 mins. The MDA content was detected by measuring absorbance at 532 nm.

### ROS level detection

Cardiomyocyte ROS level was detected by CellROX Green assay kit (Invitrogen) [27]. Briefly, CellROX Green Reagent was added to each well containing cardiomyocytes with different treatments at a concentration of 10 mmol/L and mixed vigorously. Fluorescence of CellROX was measured using a plate reader to detect the relative cardiomyocyte ROS level.

### Statistical analysis

Results are expressed as mean ± standard deviation. Statistical comparisons were made by a one-way analysis of variance followed by Bonferroni’s post-hoc analysis or unpaired Student’s t-test using GraphPad Prism 5 software (San Diego, USA). Probability values of P <0.05 were considered significant.

## Results

### Identification of DEGs in GSE173884 and GSE161827

The study was undertaken to identify possible hub genes associated with DCM progression through bioinformatics analysis and to validate the role of HMGCS2 in DCM progression using a cellular model of high glucose (HG)-induced DCM. The common DEGs between GSE173884 and GSE161827 were used for PPI network analysis. Cardiomyocyte viability and apoptosis was determined by CCK-8 and TUNEL assay, respectively; caspase-3 and-9 activity, total antioxidant, SOD activity, CAT activity, GSH content, MDA content, and ROS level were determined by respective assay kits. The expression of respective mRNAs was measured by qRT-PCR.

Firstly, DEGs from GSE173384 and GSE161827 were extracted by using GREIN-iLINCs. The results demonstrated that 231 DEGs between DCM heart of db/db mice and normal hearts of wild-type mice in GSE173384 were found; 218 DEGs between DCM hearts of four mice fed a high-fat, high-sucrose diet and normal hearts of four mice fed with control diet in GSE161827 were extracted (Figure 2(a)). Common DEGs between GSE173384 and GSE161827 were illustrated by a Venn diagram with 17 common DEGs extracted (Figure 2(b)). To explore hub genes from these common DEGs, we first constructed a PPI network of common DEGs using the STRING tool and identified 12 nodes and 17 edges in this network (Figure 2(c)). Furthermore, we used the Cytohubba tool to screen hub genes, and based on the analytic results from Cytohubba, 10 hub genes with 15 edges were found in this submodule (Figure 2(d)). Based on the literature research, we proposed that HMGCS2 may be involved in DCM and chose this hub gene for further validation studies.

**Figure 2.** Identification of DEGs between GSE173384 and GSE161827 and PPI network of common DEGs between GSE173384 and GSE161827. (a) The DEGs extracted from GSE173384 and GSE161827. (b) Common DEGs between GSE173384 and GSE161827. (c) PPI network analysis of common DEGs between GSE173384 and GSE161827. (d) Submodule network extracted from PPI network by using Cytohubba tool.

### Effects of HG on the HMGCS2 mRNA expression, cell proliferation, and apoptosis of cardiomyocytes

Cardiomyocytes were stimulated with HG or the corresponding osmotic solution, and qRT-PCR results showed that HG treatment elevated HMGCS2 mRNA expression level in cardiomyocytes compared to osmotic control group (Figure 3(a)). Consistently, HG also induced up-regulation of atrial natriuretic peptide (ANP) and brain natriuretic peptide (BNP) in cardiomyocytes compared to osmotic control group (Figure 3(b,c)). Further assays showed that HG suppressed cell viability but increased apoptosis and elevated caspase-3 and caspase-9 activities in cardiomyocytes compared to the osmotic control group (Figure 3(d-g)).

**Figure 3.** Effects of HG on the HMGCS2 mRNA expression, cell proliferation and apoptosis of cardiomyocytes. (a-c) HMGCS2(a), ANP(b) and BNP(c) mRNA expression in cardiomyocytes after treatment with blank control, osmotic control or HG was presented. (d) Cardiomyocyte viability was measured by CCK-8 assay at 72 h post-treated with blank control, osmotic control or HG. (e) Cardiomyocyte apoptosis was measured by TUNEL assay at 24 h post-treated with blank control, osmotic control or HG. (f and g) Cardiomyocyte caspase-3 and caspase-9 activities were evaluated by caspase-3 and caspase-9 activity kits at 24 h post-treated with blank control, osmotic control or HG. N = 3. Significant level was annotated as *P < 0.05, **P < 0.01 and ***P < 0.001.

### Effects of HG on cardiomyocyte inflammation and oxidative stress

Pro-inflammatory markers in cardiomyocytes after HG or osmotic solution treatment were assessed by qRT-PCR. Consistently, interleukin (IL)-1β, IL-6 and tumor necrosis factor α (TNF-α) mRNA expression were up-regulated in the HG group compared to the osmotic control group (Figure 4(a-c)). Oxidative stress was evaluated in cardiomyocytes after HG or osmotic solution treatment. HG treatment suppressed SOD, CAT, and glutathione peroxidase (GPx) mRNA expression in cardiomyocytes compared to the osmotic control group. Furthermore, HG treatment decreased total antioxidant capacity, SOD activity, CAT activity, and GSH content (Figure 4(g-j)), but increase MDA content and ROS level in cardiomyocytes compared to osmotic solution-treated cardiomyocytes (Figure 4(k,l)).

**Figure 4.** Effects of HG on inflammation and oxidative stress in cardiomyocytes. (a-c) The expression of IL-1β, IL-6 and TNF-α in cardiomyocytes after treatment with blank control, osmotic control or HG was presented. (d-f) SOD, CAT and GPx expression in cardiomyocytes after treatment with blank control, osmotic control or HG was presented. (g) Cardiomyocyte total antioxidant was determined by total antioxidant kit at 24 h post-treated with blank control, osmotic control or HG. (h-i) Cardiomyocyte SOD and CAT activity was determined by SOD and CAT activity kit, respectively, at 24 h post-treated with blank control, osmotic control or HG. (j) Cardiomyocyte GSH content was determined by GSH assay kit at 24 h post-treated with blank control, osmotic control or HG. (k) Cardiomyocyte MDA content was determined by MDA assay kit at 24 h post-treated with blank control, osmotic control or HG. (l) Cardiomyocyte ROS level was determined by ROS assay kit at 24 h post-treated with blank control, osmotic control or HG. N = 3. Significant level was annotated as *P < 0.05, **P < 0.01 and ***P < 0.001.

### Actions of HMGCS2 overexpression in cardiomyocyte proliferation and apoptosis

Actions of HMGCS2 overexpression in cardiomyocyte proliferation and apoptosis were examined. Transfection of pcDNA3.1-HMGCS2 caused a significant elevation of HMGCS2 mRNA in cardiomyocytes comparing to pcDNA3.1 transfection (Figure 5(a)). HMGCS2 overexpression also increased the ANP and BNP mRNA levels in cardiomyocytes (Figure 5(b,c)). Moreover, we examined the cell viability, apoptosis, and caspase-3 and caspase-9 activities in cardiomyocytes transfected with pcDNA3.1 or HMGCS2-overexpressing plasmids. Cardiomyocyte viability showed a significant decrease in pcDNA3.1-HMGCS2 group compared to pcDNA3.1 group (Figure 5(d)). Consistently, we found that cardiomyocyte apoptosis, caspase-3, and caspase-9 activities were increased after HMGCS2 overexpression when compared to cardiomyocytes with pcDNA3.1 transfection (Figure 5(e-g)).

**Figure 5.** Effects of HMGCS2 overexpression on cell proliferation and apoptosis of cardiomyocytes. (a-c) The expression of HMGCS2(a), ANP(b) and BNP(c) mRNA in cardiomyocytes with pcDNA3.1 or pcDNA3.1-HMGCS2 transfection was presented. (d) Cardiomyocyte viability was measured by CCK-8 assay at 72 h post-treated with pcDNA3.1 or pcDNA3.1-HMGCS2. (e) Cardiomyocyte apoptosis was measured by TUNEL assay at 24 h post-transfected with pcDNA3.1 or pcDNA3.1-HMGCS2. (f and g) Cardiomyocyte caspase-3 and caspase-9 activities were evaluated by caspase-3 and caspase-9 activity kits at 24 h post-transfected with pcDNA3.1 or pcDNA3.1-HMGCS2. N = 3. Significant level was annotated as *P < 0.05 and **P < 0.01.

### Effects of HMGCS2 on cardiomyocytes inflammation and oxidative stress

HMGCS2 overexpression elevated IL-1β, IL-6 and TNF-α expression in cardiomyocytes compared to pcDNA3.1 control (Figure 6(a-c)). The effects of HMGCS2 on oxidative stress in cardiomyocytes were further examined. The qRT-PCR assays demonstrated that HMGCS2 overexpression suppressed SOD, CAT, and GPx mRNA expression in cardiomyocytes compared to pcDNA3.1-transfected cardiomyocytes (Figure 6(d-f)). Consistently, HMGCS2 overexpression decreased total antioxidant, SOD activity, CAT activity, GSH content (Figure 6(g-j)), but increase MDA content and ROS level in cardiomyocytes compared to pcDNA3.1-transfected cardiomyocytes (Figure 6(k,l)).

**Figure 6.** Effects of HMGCS2 on inflammation and oxidative stress in cardiomyocytes. (a-c) The expression of IL-1β, IL-6 and TNF-α in cardiomyocytes with pcDNA3.1 or pcDNA3.1-HMGCS2 transfection was presented. (d-f) The expression of SOD, CAT and GPx in cardiomyocytes with pcDNA3.1 or pcDNA3.1-HMGCS2 transfection was presented. (g) Cardiomyocyte total antioxidant was determined by total antioxidant kit at 24 h post-treated with pcDNA3.1 or pcDNA3.1-HMGCS2. (h-i) Cardiomyocyte SOD and CAT activity was determined by SOD and CAT activity kit, respectively, at 24 h post-treated with pcDNA3.1 or pcDNA3.1-HMGCS2. (j) Cardiomyocyte GSH content was determined by GSH assay kit at 24 h post-treated with pcDNA3.1 or pcDNA3.1-HMGCS2. (k) Cardiomyocyte MDA content was determined by MDA assay kit at 24 h post-treated with pcDNA3.1 or pcDNA3.1-HMGCS2. (l) Cardiomyocyte ROS level was determined by ROS assay kit at 24 h post-treated with pcDNA3.1 or pcDNA3.1-HMGCS2. N = 3. Significant level was annotated as *P < 0.05.

### Actions of HMGCS2 silence on cardiomyocyte proliferation and apoptosis with HG stimulation

Effects of HMGCS2 silence on cardiomyocyte proliferation and apoptosis under HG conditions. Cardiomyocytes with HMGCS2 siRNA transfection exhibited significant down-regulation of HMGCS2 compared to si-NC transfection (Figure 7(a)). HMGCS2 silence repressed ANP and BNP mRNA expressions in HG-treated cardiomyocytes compared to the HG group (Figure 7(b,c)). CCK-8 assay revealed that HMGCS2 silence exhibited inhibitory actions on HG-treated cardiomyocyte viability compared to the HG group (Figure 7(d)). Moreover, HMGCS2 silence promoted apoptosis, caspase-3, and caspase-9 activities of cardiomyocytes compared to si-NC group (Figure 7(e-g)).

**Figure 7.** Effects of HMGCS2 silence on cardiomyocytes proliferation and apoptosis under HG conditions. (a) The expression of HMGCS2 mRNA in cardiomyocytes after treatment with si-NC or si-HMGCS2 was presented. (b and c) ANP and BNP mRNA expression in cardiomyocytes from the control, osmotic control, HG or HG + si-HMGCS2 group was shown. (d) Cardiomyocyte viability from the control, osmotic control, HG or HG + si-HMGCS2 group was determined by CCK-8 assay. (e and f) Cardiomyocyte caspase-3 and caspase-9 activities from control, osmotic control, HG or HG + si-HMGCS2 group were measured by caspase-3 and caspase-9 activity kits. N = 3. Significant level was annotated as *P < 0.05 and **P < 0.01.

### Actions of HMGCS2 silence in cardiomyocyte inflammation and oxidative stress under HG conditions

Furthermore, the actions of HMGCS2 silence in cardiomyocyte inflammation and oxidative stress under HG conditions were assessed. HMGCS2 silence decreased IL-1β, IL-6, and TNF-α mRNA expression in HG-treated cardiomyocytes compared to the HG group (Figure 8(a-c)). Further results showed that HMGCS2 silence exhibited suppressive action in SOD, CAT, and GPx mRNA expression of HG-treated cardiomyocytes compared to HG group (Figure 8(d-f)). Moreover, HMGCS2 silence attenuated HG-induced decrease in total antioxidant capacity, SOD activity, CAT activity, GSH content, and increase in MDA content and ROS level in cardiomyocytes (Figure 8(g-l)).

**Figure 8.** Actions of HMGCS2 silence on cardiomyocytes inflammation and oxidative stress under HG conditions. (a-c) IL-1β, IL-6 and TNF-α expression in cardiomyocytes from control, osmotic control, HG or HG + si-HMGCS2 was presented. (d-f) SOD, CAT and GPx expression in cardiomyocytes from control, osmotic control, HG or HG + si-HMGCS2 group was presented. (g) Cardiomyocyte total antioxidant from control, osmotic control, HG or HG + si-HMGCS2 group was presented. (h-i) Cardiomyocyte SOD and CAT activity from control, osmotic control, HG or HG + si-HMGCS2 group was presented. (j) Cardiomyocyte GSH content from control, osmotic control, HG or HG + si-HMGCS2 group was presented. (k) Cardiomyocyte MDA content from control, osmotic control, HG or HG + si-HMGCS2 group was presented. (l) Cardiomyocyte ROS level from control, osmotic control, HG or HG + si-HMGCS2 group was presented. N = 3. Significant level was annotated as *P < 0.05.

## Discussion

DCM is one of DM-related complications and progression of DCM may eventually lead to heart failure, while mechanisms related to DCM pathophysiology remain unclear [9,28,29]. This study first explored microarray datasets, including GSE173384 and GSE161827, and identified 17 common DEGs between GSE173384 and GSE161827. Further analysis of the PPI network identified nine hub genes and HMGCS2; one of the hub genes was chosen for in vitro functional analysis. The in vitro functional assays showed that HG induced up-regulation of HMGCS2, suppressed cardiomyocytes viability, enhanced apoptosis, inflammation, and oxidative stress of cardiomyocytes. Gain-of-function assays showed that HMGCS2 overexpression reduced cell viability, increased apoptosis, caspase-3/-9 activity, up-regulated IL-1β, IL-6, and TNF-α expression, decreased SOD, CAT, and GPx expression, increased MDA content and ROS level but inhibited total antioxidant activity, SOD activity, CAT activity, and GSH content in cardiomyocytes. Rescue experiments demonstrated HMGCS2 silence attenuated HG-induced decrease in cardiomyocyte viability and increase in cardiomyocyte apoptosis and oxidative stress. All in all, our study identified HMGCS2 as a hub gene in DCM pathophysiology and further functional studies indicated that HMGCS2 may aggravate DCM progression by reducing cardiomyocyte viability, increasing cardiomyocyte apoptosis, and promoting inflammation and oxidative stress in cardiomyocytes.

In GSE173384, studies performed RNA-sequencing analysis on heart tissues from the mouse DCM model, and revealed that changes in N6-methyladenosine modification contributed to DCM progression by modulating myocardial fibrosis and myocyte hypertrophy [15]. In GSE161827, Croteau et al. performed RNA sequencing analysis in the left ventricular heart tissues from the DM mice and normal mice, and the results showed that ertugliflozin could modulate the oxidative phosphorylation-related genes in the heart tissues in a DCM mouse model [30]. In our study, we identified the DEGs in the heart tissues between control mice and DCM mice and screened common DEGs that may be associated with DCM progression. Further analysis also revealed nine hub genes including HMGCS2 in the submodule. This analytical strategy has also been applied in other studies. Dong et al. performed an integrated bioinformatics analysis and revealed key candidate genes and pathways that may be associated with the protective effect of liraglutide on diabetic cardiac muscle [31]. As HMGCS2 has been found to exert important actions in the cardiomyocytes, we further selected this gene for the subsequent functional study.

The cellular model of HG-induced DCM has been widely used in exploring the molecular mechanisms of DCM. Rajesh et al. showed that the HG treatment for 48 h induced cytosolic and mitochondrial ROS production and promoted apoptosis in cardiomyocytes, which were attenuated by the cannabidiol treatment [32]. Li et al. showed that HG could induce oxidative stress and promote inflammatory response in H9C2 cardiomyocytes, which can be partially reversed by luteolin [33]. Yao et al. also demonstrated that HG treatment could promote autophagy and alleviate apoptosis in cardiomyocytes [34]. Our results showed that HG treatment suppressed cell viability, increased apoptosis, caspase-3/-9 activity, elevated IL-1β, IL-6, and TNF-α mRNA levels, reduced oxidative stress, indicating that HG could suppress cell viability, promote cell apoptosis and inflammation, and enhance oxidative stress in cardiomyocytes. More importantly, HG treatment also significantly elevated HMGCS2 levels in cardiomyocytes, suggesting that HMGCS2 may be involved in the cellular model of HG-induced DCM.

HMGCS2 is a key enzyme that controls ketone synthesis [35]. Expression and activity of HMGCS2 are regulated by several transcription factors and by posttranslational modifications including acetylation [36]. In particular, it has been reported that HMGCS2 expression was repressed by c-Myc, which is activated by the Wnt/β-catenin pathway, in colon cancer cells [36]. In human cancers, the expression level and cellular function of HMGCS2 are controversial depending on tissue types; increased expression of HMGCS2 has been observed in breast and prostate cancers, whereas diminished expression has been shown in esophageal squamous cell carcinoma, hepatocellular carcinoma, and CRC [36]. Studies also showed that HMGCS2 expression was elevated in right ventricles from patients with cardiomyopathy [37]. In addition, HMGCS2 was also elevated heart tissues from streptozotocin-induced diabetic rat [38]. Li et al. showed that exercise training could reverse lipotoxicity-induced cardiomyopathy by repressing HMGCS2 [35]. Wang et al. demonstrated that silencing of peroxisome proliferator-activated receptor-alpha alleviated myocardial injury in DCM by repressing HMGCS2 expression [39]. Sikder et al. showed that circulating HMGCS2 was elevated in the high-fat diet-induced diabetic rats [40]. Zhang et al. demonstrated that Ras/mitogen-activated protein kinase/peroxisome proliferator-activated receptor gamma inhibition could attenuate erectile dysfunction in diabetes by HMGCS2 suppression [41]. Our results showed that HMGCS2 overexpression suppressed cardiomyocyte viability, enhanced cardiomyocyte apoptosis, inflammation, and oxidative stress. On the other hand, our results further indicated that HMGCS2 silence attenuated HG-induced DCM in cardiomyocytes by increasing cell viability, while inhibiting apoptosis, inflammation, and oxidative stress.

Several limitations should be addressed in our work. First, the role of HMGCS2 has been determined in the diabetic rats, which may limit the novelty of our work. Second, HMGCS2-mediated downstream signaling pathways such as NF-κB signaling have not been examined, which may be considered in future studies. Third, the underlying mechanisms of HMGCS2-mediated apoptosis have not been fully explored, and further studies should explore the protein expression levels such as caspase-3/-9, Bax, and Bcl-2 to decipher HMGCS2-mediated cardiomyocyte apoptosis. Fourthly, the present study only determined the role of HMGCS2 in the cell model of DCM, and other hub genes identified from this study may be worthy of further investigation.

## Conclusions

In conclusion, this study identified HMGCS2 as a hub gene that may be associated with DCM progression by performing bioinformatics analysis. Further, in vitro functional studies revealed that HMGCS2 was up-regulated in HG-induced cardiomyocytes, and silence of HMGCS2 could promote cell viability, inhibit apoptosis, inflammation, and oxidative stress, which subsequently attenuated HG-induced DCM in cardiomyocytes. However, our in vitro findings should still be validated in the in vivo animal models.

## Supplementary Material

Supplemental Material

## Data Availability

All the data are available from the corresponding author.
